# Differences in Older Patients' Attitudes Toward Deprescribing at Contextual and Individual Level

**DOI:** 10.3389/fpubh.2022.795043

**Published:** 2022-02-11

**Authors:** Monika Pury Oktora, Angela Elma Edwina, Petra Denig

**Affiliations:** ^1^Department of Clinical Pharmacy and Pharmacology, University Medical Center Groningen (UMCG), University of Groningen, Groningen, Netherlands; ^2^Faculty of Science and Engineering, Medical Pharmaceutical Sciences Programme, University of Groningen, Groningen, Netherlands; ^3^Unit of Geriatrics and Gerontology, Department of Public Health and Primary Care, KU Leuven – University of Leuven, Leuven, Belgium

**Keywords:** deprescribing, older adults, polypharmacy, patient attitude, rPATD

## Abstract

**Background:**

Deprescribing requires patients' involvement and taking patients' attitudes toward deprescribing into account. To understand the observed variation in these attitudes, the influence of contextual-level factors, such as country or healthcare setting, should be taken into account.

**Methods:**

We conducted a systematic review of studies using the revised Patients' Attitudes Towards Deprescribing (rPATD) questionnaire among older adults. We searched articles in Medline and Embase up to 30 June 2021. PRISMA guideline was used for the search process and reporting. We summarized the outcomes from the rPATD and compared attitudes at study population level between high or low-middle-income countries, global regions, and healthcare settings using ANOVA testing. Correlations of the rPATD outcomes with the mean age of the study populations were tested. Associations with the rPATD outcomes at individual patient level extracted from the included studies were summarized.

**Results:**

Sixteen articles were included. Percentages of patients willing to stop medication were significantly lower in low-middle-income countries (<70% in Nepal and Malaysia) compared to high-income countries (>85% in USA, Australia, European countries). No significant differences were observed when results were compared by global region or by healthcare setting but a high willingness (>95%) was seen in the two studies conducted in an inpatient population. A higher mean age at study level was associated with a higher willingness to stop medication. At individual level, associations between patient characteristics, including demographics and education, and attitudes toward deprescribing showed inconsistent results.

**Conclusion:**

Findings about attitudes toward deprescribing are influenced by contextual factors. Future research should pay more attention to the influence of the healthcare system and setting as well as the culture on patients' attitudes.

## Introduction

Medication optimization is important for older people using multiple medicines. This includes deprescribing, which is the process of withdrawing or reducing a patient's medication in order to prevent or mitigate negative effects and improve patient outcomes (1). Deprescribing requires a patient-centered approach and involvement of the patients (2). The patients' attitudes toward their medication and deprescribing should be integrated into a shared decision-making process (3). These attitudes vary between patients and different deprescribing typologies have been described for older people with polypharmacy (4, 5). Recently, some studies have looked at individual-level factors that may explain differences in the attitudes toward deprescribing (6–8). Patient demographics, like age or sex, and a number of medications used were inconsistently associated with the patients' willingness to stop medication. Most of these studies, however, are limited by restricting the included population to certain age groups or healthcare settings. The influence of contextual-level factors, such as the healthcare system or country, was not addressed. We present a review of studies assessing patients' attitudes toward deprescribing introducing an ecological perspective to identify contextual-level next to individual-level factors that may explain differences in these attitudes, and discuss implications for future research.

## Methods

We conducted a systematic review including English-language articles published up to 30 June 2021, using the search terms “rPATD,” “attitudes toward deprescribing,” or “attitudes towards deprescribing.” The Preferred Reporting Items for Systematic Reviews and Meta-Analyses (PRISMA) guideline and checklist was used for the search process and to guide reporting. We included articles using the same instrument to prevent variation caused by the questionnaire, and chose the revised Patients' Attitudes Towards Deprescribing (rPATD) questionnaire, which has been validated and translated in several languages (9).

Two researchers independently reviewed the articles to include original studies among older adults (≥60 years) using this questionnaire. Studies adapting the rPATD questions to a specific drug or drug class were excluded. We extracted data on country, healthcare setting, study period, in/exclusion criteria, response rate, and patient characteristics. Countries were grouped in global regions. Healthcare settings were classified as [1] primary care or home dwelling, [2] outpatient care provided by hospital, [3] secondary or inpatient hospital care, [4] nursing homes, and [5] mixed. Next, we extracted the outcomes from the rPATD. In particular, we extracted percentages of patients willing to stop medication, and satisfied with their medication. Furthermore, we extracted results regarding the four factors covered by the rPATD: “burden of medication,” “appropriateness of medication,” “concerns about stopping,” and “involvement in decision making.” Means with standard deviations or median with interquartile ranges were summarized. One study presented factor scores on a scale up to 100 (10), which we divided by 20 to represent the original scale up to 5. For one study that presented “inappropriateness” without carrying out the inverse scoring (11), we reversed the scores and reported associations. We tested for differences at study level in (a) willingness to stop medication, (b) satisfaction with medication, and (c) the four rPATD factors using ANOVA, comparing global regions (USA, Europe, Australia, Asia, Africa), high-income versus low-middle-income countries (OECD classification), and healthcare settings (primary care, outpatient, inpatient, nursing home). For studies reporting outcomes among subpopulations from different healthcare settings, the data were tested at this level. We also tested for associations of the rPATD outcomes with the mean or median age of the study (sub)population using Pearson Correlation. Expecting sample sizes >25, the median was considered as the best estimator for the mean (12). All tests were 2-sided and conducted with SPSS Statistics v23.0 for Windows. Finally, we extracted and summarized data from the studies testing for associations with the rPATD outcomes at individual level regarding the patients' age, sex, educational level, number of drugs used, and healthcare setting.

## Results

We identified 198 titles and abstracts and excluded 182 for not meeting our inclusion criteria, resulting in 16 included articles referring to 14 data collections. The included studies were conducted in 11 different countries and recruited patients from all possible healthcare settings. The median number of drugs taken by the patients ranged from three to 10.

### Differences in Attitudes at Contextual Level

In 13 studies reporting on willingness, the majority of older adults were willing to have one or more of their regular medications stopped if their physician said it is possible, with percentages ranging from 57 to 97% (Figure 1A). Of note, the populations with the lowest percentages of 57 and 68% had high percentages of 19 and 24% of patients being unsure about their willingness (6, 13). In other studies, these percentages of being unsure were <10% (10, 14–18). A higher willingness was observed in high-income countries as compared to low-middle-income countries (*n* = 12, ANOVA, F 15.426, *p*-value 0.002), with highest percentages in the USA (average 91%) (16, 19), followed by Australia (88%) (18), and European countries (average 87%) (8, 10, 14, 15, 17, 20, 21). Intermediate precentages were seen in Singapore (83%) and Ethiopia (82%) (11, 22), whereas the lowest percentages were observed in Nepal and Malaysia (57%, 68%) (6, 13). There was no significant difference in willingness between healthcare settings, although the highest willingness percentages (>95%) were seen in the two studies conducted in inpatient care (Figure 1A) (10, 20). The willingness was not significantly different between global regions. Finally, a higher average age of the study (sub)population was associated with a higher willingness (n = 16, Pearson Correlation, 0.685, *p*-value 0.003).

**Figure 1:** **(A)** Satisfaction and willingness scores across study (sub)populations. Bars are presented with setting, country, and mean age of study (sub)population in the labels, including the reference number in superscript. DEN, Denmark; UK, United Kingdom; USA, United States of America; AUS, Australia; NL, Netherlands; SWI, Switzerland; SIN, Singapore; SP, Spain; ETH, Ethiopia; MLY, Malaysia; NEP, Nepal; NA, not assessed; PC/NH, primary care/nursing home. **(B)** rPATD factor scores across study (sub)populations. Bars are presented with setting, country and mean age of study (sub)population in the labels, including the reference number in superscript. rPATD, revised Patients' Attitudes Towards Deprescribing; No PIM/PIM, subgroups without or with potentially inappropriate medication subgroups; SWI, Switzerland; NL, Netherlands; MLY, Malaysia; SIN, Singapore; DEN, Denmark; USA, United States of America; NEP, Nepal.

In 11 studies reporting on satisfaction, the majority of older adults were satisfied with their medication, with percentages ranging from 69 to 97% (Figure 1A). These percentages did not significantly differ between healthcare settings, economic level of the countries, and was also not associated with the mean age of the study population. There was a difference in satisfaction between the global regions (*n* = 10, ANOVA, F 4.639, *p*-value 0.043). The highest percentages of satisfaction were seen in Africa (92%) and Europe (average 89%) and the lowest in the USA (69%) (8, 10, 14–17, 20, 22).

In 10 studies presenting the mean or median rPATD factor scores, “appropriateness” ranged from 2.8 to 3.8, “concerns” from 1.6 to 2.8, “burden” from 2.1 to 3.1, and “involvement” from 3.2 to 4.8 (Figure 1B). These factors were not significantly associated with the economic level of the country, healthcare setting, nor global region. A higher aged study population was associated with less concerns (*n* = 10, Pearson Correlation, −0.696, *p*-value 0.025) and less burden (*n* = 10, Pearson Correlation, −0.677, *p*-value 0.031).

### Differences in Attitudes at Individual Patient Level

In seven studies, age was not significantly associated with any of the rPATD outcomes (8, 10, 11, 14, 17–19), whereas inconsistent findings were observed in three studies (6, 13, 23) (Table 1). A higher age was associated with less willingness in one study (13) but more willingness in another study (6). Sex was not associated with any of the rPATD outcomes in nine studies (6, 8, 10, 13, 14, 17–19, 23). In one study, males showed lower appropriateness but higher satisfaction and involvement scores (11). A higher number of drugs was associated with more willingness in two studies (11, 19), but not associated with willingness in four studies (6, 8, 14, 18). Furthermore, a higher number of drugs was associated with higher burden scores in four studies (10, 11, 14, 23), whereas an opposite association was seen in one study (6). For educational level, a positive association was found with willingness in two studies (8, 18), a negative association in one study (6) and no association in another study (19). Only two studies tested for the influence of setting, indicating that patients recruited in outpatient setting may have higher willingness as compared to a primary care setting (11), but inconsistent results were observed for involvement scores (10, 11).

**Table 1:** Characteristics associated with the two global questions and four factors outcomes from the revised Patients' Attitudes Towards Deprescribing (rPATD) questionnaire.

**References**	**Analysis**	**Outcomes rPATD**	**Non-significant characteristics**	**Significant characteristics**
Crutzen et al. (14)	Linear and ordinal logistic regression	Satisfaction	Age; sex; number of drugs (≤5, 5–10, >10)	–
		Willingness	Age; sex; number of drugs (≤5, 5–10, >10)	–
		Appropriateness	Age; sex; number of drugs (≤5, 5–10, >10)	–
		Concerns	Age; sex; number of drugs (≤5, 5–10, >10)	–
		Burden	Age; sex	Number of drugs (>10), beta-coefficient 0.41
		Involvement	Age; sex; number of drugs	–
Kua et al. (6)	Spearman's correlations (univariate)	Willingness	Sex; number of drugs	Age (60–74 or ≥75), correlation 0.131 Education (primary, secondary, higher), correlation −0.158
		Appropriateness	Age (60–74 or ≥75); sex; education (primary, secondary, higher)	Number of drugs, correlation −0.219
		Concerns	Age (60-74 or ≥75); sex	Education (primary, secondary, higher), correlation 0.118 Number of drugs, correlation −0.191
		Burden	Age (60–74 or ≥75); sex; education (primary, secondary, higher)	Number of drugs, correlation −0.344
		Involvement	Sex; number of drugs	Age (60–74 or ≥75), correlation 0.267 Education (primary, secondary, higher), correlation −0.211
Kua et al. (11)	Mann-Whitney U; Kruskal-Wallis test (univariate)	Satisfaction	Age (<80 vs. 80+); education; setting (outpatient vs. primary care)	Sex, male > female Number of drugs, ≤5 > more than 10
		Willingness	Age (<80 vs. 80+); sex; education	Setting, outpatient > primary care Number of drugs, more > less (≤5, 5–10, >10)
		Appropriateness	Age (<80 vs. 80+); education	Sex, female > male Number of drugs, less > more (≤5, 5–10, >10) Setting, community hospital < other hospital and community pharmacy
		Concerns	Age (<80 vs. 80+); sex; number of drugs (≤5, 5–10, >10); setting (outpatient vs. primary care)	Education, direction not clear
		Burden	Age (<80 vs. 80+); sex; education; setting (outpatient vs. primary care)	Number of drugs, more > less (≤5, 5–10, >10)
		Involvement	Age (<80 vs. 80+); number of drugs (≤5, 5–10, >10)	Sex, male > female Education, higher > lower Setting, outpatient > primary care
Lundby et al. (10)	Quantile regression (univariate)	Appropriateness	Age (<80 vs. 80+); sex; setting (inpatient, outpatient, nursing home)	Number of drugs, less > more (≤5, 5–9, ≥10)
		Concerns	Age (<80 vs. 80+); sex; setting (inpatient, outpatient, nursing home)	Number of drugs, more > less (≤5, 5–9, ≥10)
		Burden	Age (<80 vs. 80+); sex; setting (inpatient, outpatient, nursing home)	Number of drugs, more > less (≤5, 5-9, ≥10)
		Involvement	Age (<80 vs. 80+); sex; number of drugs (≤5, 5–9, ≥10)	Setting, outpatient > nursing home and inpatient
Omar et al. (23)	Spearman correlations (univariate)	Appropriateness	Sex	Age, correlation −0.174 Number of drugs, correlation −0.176
		Concerns	Age; sex; number of drugs	–
		Burden	Sex	Age, correlation 0.183 Number of drugs, correlation 0.271
		Involvement	Age; sex; number of drugs	–
Reeve et al. (19)	Logistic regression	Willingness	Age (65–74, 75–84, ≥85); sex; education (low, medium, high)	Number of drugs (≥6 drugs), aOR 2.90 (adjusted also for race, health, number of chronic medical conditions)
Reeve et al. (18)	Logistic regression	Willingness	Age (65–74 vs. ≥75); sex, number of drugs (≥6 drugs)	Education (English as first language), aOR 3.78 (adjusted also for burden, appropriateness, concerns, autonomy, health, goal of care, insurance)
Rozsnyai et al. (8)	Logistic regression	Willingness	Age; sex; number of drugs	Education, high > low, OR 3.28 (adjusted also for living alone, self-management of medication)
Serrano Gimenez et al. (17)	Odds ratio (univariate)	Satisfaction	Age (<70 vs. ≥70); sex; education (low vs. other)	Polypharmacy, >6 drugs, OR 1.33
Shrestha et al. (13)	Logistic regression	Willingness	Sex; education (up to high school), number of drugs (≥5 drugs)	Age, OR 0.95 (adjusted for concern about stopping)

## Discussion

### Principal Findings

Looking at contextual level, we observed that populations from low-middle-income countries were less willing to stop medication than those from high-income countries. The highest average willingness scores were seen in inpatient settings. At population level, a higher average age was associated with a higher willingness but usually no associations with age were observed at individual level. At individual level, a higher number of drugs was sometimes associated with more willingness and higher burden scores. In general, the patients' sex or education were not associated with their attitudes toward deprescribing.

Recent meta-analyses showed pooled proportions of willingness to stop medication between 84 and 88% (24, 25). We observed no differences when studies were compared by global region, confirming previous results (24). Possibly such regions are too heterogeneous to identify differences related to the healthcare system or culture. In our review, the lowest percentages of willingness were seen in Malaysia and Nepal (6, 13), whereas patients from high-income countries showed a higher willingness. So far, there have been few studies from low-middle-income countries and more studies are needed to strengthen our finding and identify underlying mechanisms. We noticed that both studies with low percentages of willingness showed high percentages of patients being unsure about this. It could be that in these countries there are less initiatives to optimize medication and involve patients in such processes (26, 27). Previously, it was found that the Southeast-Asian hierarchical culture and one-way communication style of healthcare professionals inhibits patients to ask questions (28).

Although we did not see any significant associations between the healthcare setting and attitudes toward deprescribing, high willingness scores were seen in both studies conducted in a geriatric ward setting (10, 20). A *post-hoc* analysis showed a significant difference in willingness between this setting as compared to the combined other settings (*n* = 13, ANOVA, F 4.896, *p*-value 0.045). This suggests that when patients are admitted to a geriatric ward this can be a good opportunity to initiate deprescribing. Of note, combining patients recruited at hospital wards with those recruited at outpatient clinics as “hospital setting” or “secondary/tertiary care,” as done previously (24, 25), may lead to loss of relevant information. One study in our review observed that patients in a primary care setting were less willing to stop medication as compared to an outpatient hospital setting (11). More studies are needed comparing patients recruited from different healthcare settings to ascertain which settings require more effort when involving patients to initiate deprescribing.

When looking at individual patient characteristics, it is still not clear which factors should be taken into account when implementing deprescribing. Patients' sex appears to be irrelevant but findings regarding associations with age, number of drugs and education are inconsistent, in line with findings from previous reviews (24, 25). To gain better insight, more attention should be paid to the influence of the selected study population. For example, we observed a positive association between age and willingness at study level, and this was also observed within one study that included relatively young patients, comparing the group from 60–74 to ≥75 years (6). Most studies observing no association compared older age groups (8, 10, 11, 14, 17–19), indicating that differences among patients of ≥65 years are less relevant. Regarding number of drugs and education, the context should be taken into account. There was a wide range in the median number of drugs taken by patients, possibly related to the healthcare setting where patients were recruited. Testing for associations with the number of drugs within a population using on average three drugs (6) is likely to give different results then in populations using on average five drugs (11). Regarding educational level, a higher education was related to more willingness to stop medication in the USA and Switzerland and less willingness in Malaysia (6, 8, 18). Differences in overall educational level of the included population might explain such contradictory findings.

### Strengths and Limitations

All review steps were conducted by two people, following rules for conducting systematic reviews. We included studies using the same questionnaire to assess attitudes toward deprescribing, thereby reducing the chance that observed differences might be caused by the questionnaire used. As a consequence, studies using the older PATD were not included. We grouped healthcare settings in four groups but the information about the setting was sometimes limited or difficult to interpret. Particularly related to the outpatient care, quite different outpatient clinics and acute care facilities were grouped together. Furthermore, the number of studies we could include in the analysis at contextual level was rather small, which limits the power for significant findings. Finally, our analysis on mean age should be interpreted in the light of its ecological fallacy.

## Conclusion

Research findings about attitudes toward deprescribing are influenced by contextual factors partly inherent to the inclusion criteria of the study population. Future research should pay more attention to the influence of context, such as the healthcare system and setting as well as the communication culture on patients' attitudes toward deprescribing. More cross-cultural, and cross-setting studies are needed that allow for direct comparisons.

## Author Contributions

MO, AE, and PD designed the study concept and search strategy. MO and AE conducted the literature search, screened the identified articles, extracted data from eligible articles, and drafted the manuscript. PD checked eligibility, data extractions, supervised the research, and edited the manuscript. MO and PD analyzed and interpreted data. All authors read the final version and approved submission and agreed to be accountable for all aspects of the work.

## Funding

MO reports grants (scholarship) to support of her Ph.D. program from Indonesia Endowment Fund for Education (LPDP) during the conduct of the study.

## Conflict of Interest

The authors declare that the research was conducted in the absence of any commercial or financial relationships that could be construed as a potential conflict of interest.

## Publisher's Note

All claims expressed in this article are solely those of the authors and do not necessarily represent those of their affiliated organizations, or those of the publisher, the editors and the reviewers. Any product that may be evaluated in this article, or claim that may be made by its manufacturer, is not guaranteed or endorsed by the publisher.
